This article has been retracted.

# Loss of PDEF, a prostate-derived Ets factor is associated with aggressive phenotype of prostate cancer: Regulation of MMP 9 by PDEF

**DOI:** 10.1186/1476-4598-9-148

**Published:** 2010-06-15

**Authors:** Thomas R Johnson, Sweaty Koul, Binod Kumar, Lakshmipathi Khandrika, Sarah Venezia, Paul D Maroni, Randall B Meacham, Hari K Koul

**Affiliations:** 1 Program in Urosciences, Division of Urology-Department of Surgery, University of Colorado Denver School of Medicine, Denver Veterans Administrative Medical Center, and University of Colorado Comprehensive Cancer Center, Building P15 or RC2, C-317, 12700 E 19th Avenue, Aurora, CO 80045, USA

## Abstract

**Background:**

Prostate-derived Ets factor (PDEF) is expressed in tissues of high epithelial content including prostate, although its precise function has not been fully established. Conventional therapies produce a high rate of cure for patients with localized prostate cancer, but there is, at present, no effective treatment for intervention in metastatic prostate cancer. These facts underline the need to develop new approaches for early diagnosis of aggressive prostate cancer patients, and mechanism based anti-metastasis therapies that will improve the outlook for hormone-refractory prostate cancer. In this study we evaluated role of prostate-derived Ets factor (PDEF) in prostate cancer.

**Results:**

We observed decreased PDEF expression in prostate cancer cell lines correlated with increased aggressive phenotype, and complete loss of PDEF protein in metastatic prostate cancer cell lines. Loss of PDEF expression was confirmed in high Gleason Grade prostate cancer samples by immuno-histochemical methods. Reintroduction of PDEF profoundly affected cell behavior leading to less invasive phenotypes in three dimensional cultures. In addition, PDEF expressing cells had altered cell morphology, decreased FAK phosphorylation and decreased colony formation, cell migration, and cellular invasiveness. In contrast PDEF knockdown resulted in increased migration and invasion as well as clonogenic activity. Our results also demonstrated that PDEF downregulated MMP9 promoter activity, suppressed MMP9 mRNA expression, and resulted in loss of MMP9 activity in prostate cancer cells. These results suggested that loss of PDEF might be associated with increased MMP9 expression and activity in aggressive prostate cancer. To confirm results we investigated MMP9 expression in clinical samples of prostate cancer. Results of these studies show increased MMP9 expression correlated with advanced Gleason grade. Taken together our results demonstrate decreased PDEF expression and increased MMP9 expression during the transition to aggressive prostate cancer.

**Conclusions:**

These studies demonstrate for the first time negative regulation of MMP9 expression by PDEF, and that PDEF expression was lost in aggressive prostate cancer and was inversely associated with MMP9 expression in clinical samples of prostate cancer. Based on these exciting results, we propose that loss of PDEF along with increased MMP9 expression should serve as novel markers for early detection of aggressive prostate cancer.

## Background

Prostate cancer is the second leading cause of cancer death in men. In the United States alone, 192,280 new cases of prostate cancers were diagnosed in 2009 and among them around 27,360 deaths occurred. One of the biggest challenges we face in prostate cancer is determining if the cancer is aggressive. Conventional therapies produce a high rate of cure for patients with localized prostate cancer, but there is no cure once the disease has spread beyond the prostate. Reduction in serum prostate-specific antigen (PSA) levels has been proposed as an endpoint biomarker for human prostate cancer intervention. However, despite being the mainstay of prostate cancer detection, the value of PSA screening is still debated. In particular, there is a growing concern regarding the over diagnosis of potentially indolent disease [1]. Therefore, there remains an urgent need for more accurate biomarkers to diagnose aggressive prostate cancer. Thus, identification of new molecular markers/targets for aggressive prostate cancer is important in order to improve early detection of the aggressive disease and to develop new therapeutic regimens.

Progression of prostate cancer from focal, androgen-dependent lesions to androgen-independent, metastatic cancer requires deregulation of growth control, invasiveness and cell motility. Abundant evidence demonstrates roles for Ets transcription factors in many cancers including prostate. Prostate-derived Ets factor (PDEF), first described nine years ago as preferentially binding to the noncanonical Ets core sequence GGAT [2], has recently received considerable attention due to its potential importance in regulating cell motility and invasion [3-5]. Recently, proteomic analysis of PDEF overexpressing cells revealed 286 proteins in the PDEF-associated protein complex in breast cancer [6]. Thus interaction of PDEF with other partner proteins could help in finding their role in maintenance of malignant phenotype. Published literature concerning experimental manipulation of PDEF expression is paradoxical and limited to tissues of high epithelial content, notably prostate, breast, ovary and colon [7,8]. PDEF expression has been both positively [3,9] and negatively [10] correlated with breast cancer grade at mRNA or protein levels. It is important to note that PDEF mRNA and protein levels do not always correlate, which may have led to different conclusions in some of the studies examining PDEF expression in primary tumors. Turner et al. [4] found that introducing PDEF into invasive breast cancer cell lines reduced their invading ability. Similarly, siRNA-mediated knockdown of PDEF in MCF7 cells increased their ability to migrate in the Transwell assay. Besides its role in cancer metastasis, PDEF expression was also correlated with changes in the actin cytoskeleton and focal adhesion localization, and loss of cellular polarity. Ghadersohi et al. [10] silenced PDEF expression in MCF7 cells, and found that such cells showed greatly accelerated xenograft tumor formation in SCID mice. By contrast, Gunawardane et al. [3] showed that increasing expression of PDEF increased their ability to migrate in a Transwell assay and stimulated colony formation in soft agar. This group also identified a canonical MAP kinase phosphorylation site at T50 (PAT_50_P) and showed that mutation to alanine at this site abolished all the effects they observed. To date there are few data available formally correlating PDEF expression in maintenance of prostate malignant phenotype. Two published studies, one with a prostate cancer cell-line [5] and another with clinical samples from prostate [11] reached opposite conclusions with respect to the role of PDEF in prostate cancer. Clearly additional studies are necessary to evaluate role of PDEF in prostate cancer biology.

In the current studies, we report here that PDEF expression is lost, whereas MMP9 expression increased with the aggressive behavior of prostate cancer. Overexpression of PDEF in PC3 cells strongly inhibits colony formation, cell migration and invasion, and increased cell adherence. Furthermore, re-introduction of PDEF in PC3 cells led to changes in actin cytoskeleton, altered focal adhesion kinase activity, and reestablished cell polarity in these cultures as indicated by induction of less invasive spheroid-like structures in three-dimensional culture, Moreover, PDEF expression downregulates MMP9 expression, and its promoter activity in PC3 cells. Thus, consideration of both PDEF and MMP9 may have a better prognosis value for determining the aggressive phenotype of prostate cancer.

## Materials and methods

### Constructs and cell lines

All cell lines (PC3, LNCaP, and C4-2B) were purchased from ATCC and maintained according to ATCC guidelines. Phoenix cells were grown in DMEM containing 10% fetal bovine serum. FLAG tag antibody was purchased from Sigma (St. Louis, USA). PDEF and phospho FAK antibodies were from Santa Cruz Biotechnology (CA, USA). PDEF was cloned from PC3 cDNA with an amino-terminal FLAG tag, and inserted into retroviral vectors pBABE and the bicistronic vector QCXIX (Clontech). The latter vector was modified to contain a wild-type internal ribosome entry site to increase expression from the second multiple cloning site, into which G418 resistance was cloned. Mutations were created using the Quick-Change kit (Stratagene) according to the manufacturer's instructions. Oligonucleotide primers for PCR were purchased from Integrated DNA Technologies.

### Retrovirus production and infection

Phoenix cells were transfected with 2 μg DNA using Effectene (Qiagen) according to the manufacturer's instructions, and infection was followed according to Phoenix™ Retrovirus Expression System (Orbigen Inc.). After infection, cells were trypsinized, transferred to 150 mm dishes, and subjected to puromycin or G418 selection after 48 h incubation.

### Thymidine incorporation

1 × 10^5 ^cells/well were plated in 12-well plates. 48 h later, cells were exposed to medium containing1-3 μCi/ml ^3^H-thymidine (Perkin Elmer) and incubated for 4 h. After 2 washes with cold PBS, cells were fixed in cold methanol for 5 min followed by an additional methanol wash. Cells were solubilized in 0.1% SDS/0.2 M NaOH and radioactivity determined.

### Anchorage independent growth, motility, invasion and attachment assays

Growth in soft agar was performed as described previously [12]. Invasiveness was determined by the method of Repesh LA [13]. Cell migration through Transwell membranes was performed identically, but without the use of Matrigel. Wound healing assays were performed by making a cruciform scratch in a confluent monolayer of cells. Cells were washed, the medium replaced with serum-free medium, and incubated for 48-72 h. Cells were fixed with methanol, stained with Giemsa, and photographed.

Attachment assays were performed essentially by the method of Turner et al. [4] using 96-well plates pretreated overnight with fibronectin, Matrigel, or bovine serum albumin at concentrations of 50 ng/ml, 100 ng/ml, and 10 mg/ml respectively.

### Immunohistochemistry for PDEF and MMP9 expression on prostate tissue array slides

Tissue microarray slides containing 9 normal and 40 prostate cancer samples of varying pathological grade were obtained from Imgenex Corporation, San Diego, CA, 92121. Immuno histochemistry for PDEF and MMP9 was performed using the avidin-biotin complex method previously described by Hsu et al. [14]. Expression of PDEF and MMP9 were evaluated by analysis of microscopic scans of each tissue. Expression was considered high if greater than 60% of the scanned area scored positive, while expression was considered moderate if 40-60% area scored positive, and expression was considered low if less than 40% area scored positive.

### Reverse transcription PCR

Total RNA was extracted using RNEasy mini kit (Qiagen). 1 μg of RNA was used to prepare cDNA using iScript second strand cDNA synthesis kit (Bio-Rad). 100 ng of synthesized cDNA was used for RT-PCR using forward 5-TTGACAGCGACAAGAAGTGG-3 and reverse 5-TCACGTCGTCCTTATGCAAG-3 for MMP9, forward 5-ACCACAGTCCATGCCATCAC-3 and reverse 5-TCCACCACCCTGTTGCTGTA-3 for GAPDH. Transcripts were separated by agarose gel electrophoresis.

### Reporter assay

Cells were transfected with 1 μg of MMP9 luciferase reporter vector along with 10 ng of Renilla luciferase expression plasmid using Effectene (Qiagen, Valencia, CA) according to manufacturer's instructions. Luciferase activity was measured using the Dual luciferase kit (Promega Corporation, Madison, WI) with Monolight 2010 Luminometer (Analytical Luminescence laboratory, San Diego, CA).

### MMP Zymography

Zymogram for MMP9 activity was performed according to Bernhard and Muschel [15] using conditioned medium.

### Three dimensional cell culture

PDEF overexpressing PC3 cells and respective vector control cells were grown in growth factor reduced Matrigel for 10-12 days and then immunofluorescence staining was performed according to Debnath et al. [16]

### Morphology studies

Cell morphology was done on glass chamber slides by immunofluorescence method. Vector control and PDEF expressing cells were seeded on multi-chamber slide, fixed with 4% formalin, permeabilized with 0.1% Triton-X-100, blocked in 2% BSA, and change in actin cytoskeleton was examined by phalloidin staining as per the manufacturer's instructions (Molecular Probes, Eugene, OR). Pictures were taken using Spin Disc Olympus confocal microscope.

### Western Blot analysis

Electrophoresis and blotting were performed as described previously [17].

### Statistical analysis

Statistical analyses for tissue culture studies were performed using two-dimensional two sample variance T-tests; For data from clinical specimens, statistical analysis was performed using MANN - WHITNEY U: exact test. p ≤ 0.05 was considered significant.

## Results

### PDEF expression is reduced during the transition from low grade to high grade prostate cancer

PDEF expression was evaluated by immunohistochemical examination in tissue microarray slides containing 40 cores of prostate cancer and 9 cores of normal prostate. Results presented in Figure 1 show that PDEF protein expression is downregulated during the transition to aggressive prostate cancer. As shown in Figure. 1A, high levels of PDEF protein are present in normal prostate epithelial cells as well as early stage prostate cancer. However, in high grade prostate cancer PDEF protein is significantly decreased. Significant reduction in PDEF expression was observed in all cores of prostate tumor tissue with high Gleason grade (Gleason score greater than 7) as compared to normal prostate tissue as well as low grade prostate cancer (Gleason score of 7 or below). Moreover, PDEF protein levels showed graded decrease with increase in pathologically confirmed aggressive disease. Our results show that while 59 ± 3.6% tissue scored positive for PDEF in low to moderate grade (Gleason 6 & 7) prostate cancer, and 33 ± 3.3% of the tissue scored positive for PDEF in moderately high grade (Gleason 8) tumor, there was little or no expression of PDEF in very high grade (Gleason 9 & 10) prostate cancer(Figure. 1B). Antibody specificity for these assays was determined by Immunofluorescence and Western blot analysis using cells with and without PDEF expression (Figure S1, Additional file 1). In addition to clinical samples, we also evaluated PDEF protein expression in established prostate cancer cell lines with low to high aggressive behavior. These results presented in Figure 1C show that PDEF is expressed in LNCaP cells (a less aggressive prostate cancer cell line). However, PDEF expression is reduced in more aggressive lineages of LNCaP cells (C4-2 and C4-2B). Moreover, PDEF expression is completely lost in two widely used aggressive prostate cancer cells (DU145 and PC3 cells). Taken together, results of these studies demonstrate that PDEF expression is decreased or lost in prostate cancer cells with aggressive phenotype, and provide novel insights into the characteristics of PDEF protein expression in progression of prostate cancers. Absence of PDEF protein expression in PC3 cells in our studies is in apparent disagreement with previous report [5] that showed PDEF expression in PC3 cells,. This discrepancy could result from several causes: First, the antibody used in [5] could be more sensitive, such that they were able to detect even negligible amounts of PDEF. Second PC3 cells change over various passages of culture and media conditions, which could explain the differences.

**Figure 1:** **PDEF protein expression in human prostate tissues and prostate cancer cell lines**. ***A***, Representative photo-micrographs of Immuno-histochemical analysis of PDEF expression using prostate tissue micro-array slides (containing both normal and tumor samples of different grades) performed as described in Materials and Methods. ***B***, Quantification of percentage staining for PDEF. ***C***, Representative image showing Western blot analysis on prostate cancer cell lines using anti-PDEF antibody (left panel), and quantitation of the same data (right panel).

### Re-introduction of PDEF inhibited directional migration, decreased cell migration and anchorage independent growth in prostate cancer cells

To examine the effects of PDEF expression on cell motility, PC3 cells transduced with PDEF or mutant PDEF T50A, or vector alone were assayed for their ability to migrate through Transwell membranes as described in materials and methods. Results presented in Figure 2A indicate that both wild-type and mutant PDEF-transduced cells were significantly inhibited in their ability to migrate through Transwell pores. We also subjected cells to an assay for persistence migratory directionality (in vitro wound healing, Figure. 2B). Expression of either PDEF or the T50A mutant inhibited the ability of PC3 cells to fill in gaps in a monolayer compared to vector alone. These results demonstrated that PDEF significantly interfered with ability of cells to maintain migratory phenotype.

**Figure 2:** **Effect of re-introduction of PDEF on directional migration, trans-well migration and anchorage independent growth in prostate cancer cells**. ***A***, Migration of PC3 cells expressing PDEF or PDEF T50A through Transwell membranes as described in Materials and Methods. ***B***, PDEF overexpression decreases directional cell migration (*in vitro *wound healing migration of these cells). ***C***, Representative photomicrographs from experiments testing colony formation as described in Materials and Methods. ***D***, ^3^H-thymidine incorporation in PC3 PDEF overexpressing cells measured as described in Materials and Methods. ***E***, Relative expression level of PDEF in these cell lines. Asterisks indicate significance levels of p < 0.05 with respect to controls.

We next examined the effects of PDEF overexpression on the ability of PC3 cells to form colonies in soft agar. Expression of either PDEF or the T50A mutant equally inhibited the ability of PC3 cells to form colonies in soft agar (Figure. 2C) compared to vector alone.

To address the possibility that altered cell proliferation contributed to the results of these assays, we measured DNA synthesis (^3^H-thymidine incorporation) in control and PDEF transfected PC3. Results of these studies (Figure. 2D) show that decreased clonogenic activity following PDEF expression was not a consequence of decreased DNA synthesis. These results demonstrated that PDEF expression decreased clonogenic ability of the cells independent of DNA synthesis. Moreover, in sharp contrast to the effects of PDEF on anchorage independent growth, PDEF expression did not significantly affect anchorage dependent growth of prostate cancer cells in culture (data not shown).

### PDEF expression resulted in increased cell adhesion, altered cell morphology and decreased focal adhesion kinase activity in prostate cancer cells

Immunofluorescence studies of PDEF expressing cells showed a rounded area of cleared fluorescence rather than elongated track as seen on invasive vector control cells (Figure. 3A). These results indicated that PDEF expression resulted in alterations to actin cytoskeleton and altered cell morphology. FAK is a non-receptor protein tyrosine kinase, associated with supramolecular focal adhesion complexes. Focal adhesion complex assembly and disassembly are critical for cell attachment and movement [18]. The lack of morphologic polarity in PDEF expressing cells as shown in Figure 3A raised the possibility that PDEF may affect adhesion complex formation. Moreover, in previous studies we observed that FAK was non-phosphorylated in adherent cultures and FAK phosphorylation was increased in suspension culture [19]. Therefore, we evaluated the effects of re-introduction of PDEF in PC3 cells on FAK phosphorylation in PC3 cells in suspension cultures. Results of these studies revealed a significant reduction in FAK phosphorylation in PDEF expressing cells grown in suspension culture (Figure. 3B). These results demonstrated that PDEF expression in PC3 cells resulted in decreased FAK activity, suggesting decreased focal adhesion formation.

**Figure 3:** **Effects of PDEF expression in prostate cancer cells on cell morphology, FAK phosphorylation and attachment to specific substrates**. ***A***, Phalloidin staining of actin cytoskeleton in PDEF expressing and vector control cells. ***B***, Decreased phophorylation of FAK in PDEF expressing cells growing in suspension culture. ***C***, Representative photomicrographs from experiments testing attachment of PC3 cell expressing PDEF to either BSA or fibronectin or matrigel-treated plastic surface as described in Material and Methods; and quantitation of these data. Asterisks indicate significance levels of p < 0.05 with respect to controls.

Focal adhesion formation and its interaction with the ECM play a central role in migration and invasion, since increased adhesion makes cells less motile. To examine this possibility, we directly measured the effects of PDEF expression on adhesion of PC3 cells to various ECM substrates. For these studies, PC3 cells transfected with PDEF or vector alone were assayed for their ability to attach to fibronectin or Matrigel-coated plastic surfaces. Results presented in Figure 3C indicate that attachment of PDEF-expressing cells to fibronectin-coated, Matrigel-coated, or control (BSA treated) plastic was significantly increased compared to vector-transduced cells. These results are in contrast to the effects of PDEF in breast cancer cells, where PDEF was shown to decrease adhesion of the cells to fibronectin and matrigel [4]. Taken together, these results suggest that PDEF mediated inhibition of migration may occur through cytoskeleton disorganization and ECM interaction.

### PDEF decreased invasion and inhibited expression of matrix metalloproteinase-9 (MMP9) in prostate cancer cells

To test the effects of PDEF on cell invasion, we examined the effects of PDEF expression on the ability of PC3 cells to invade simulated basement membrane *in vitro*, a phenotype correlated with aggressive behavior. Results presented in Figure 4A indicate that expression of either PDEF or the T50A mutant inhibited the ability of PC3 cells to invade through Matrigel compared with vector transfected control cells. In addition to transfection of PC3 cells with PDEF, we also performed complementary RNA interference (RNAi) experiments to reduce the endogenous PDEF expression in prostate cancer cells that express PDEF (LNCaP and C4-2B cells), and directly evaluated the effects of decreased PDEF levels on invasion and clonogenic activity of these cells. Results presented in Figure S2, Additional file 1 demonstrated that SiRNA mediated knock-down of PDEF in these cells resulted in an increased ability to form colonies in soft agar and increased invasion through Matrigel basement membrane. Taken together with rest of the results these studies suggest that PDEF may play an important role in prostate cancer metastasis.

**Figure 4:** **Effect of PDEF on invasion through Matrigel Matrix and MMP9 mRNA expression, MMP9 promoter activity and MMP9 enzymatic activity of prostate cancer cells**. ***A***, Invasion of PC3 cells expressing PDEF or PDEF T50A through Transwell membranes as described in Methods. ***B***, RT-PCR showing MMP9 mRNA (left panel) and MMP9 enzymatic activity using gelatin Zymography (Right panel) was performed to determine the level of active MMP9. ***C***, MMP9 promoter activity as determined by Luciferase reporter assay. ***D***, Invasion of PC3 cells through a basement membrane matrix after blocking MMP9 using antibodies or overexpressing PDEF. Asterisks indicate significance levels of p < 0.05 with respect to controls.

Matrix metalloproteinases (MMPs) are a family of enzymes whose function primarily relates to degradation of extracellular matrix proteins, and are necessary for cell invasion. Moreover increased MMP activity has been associated with tumor metastasis. In our *in vitro *studies we observed that only MMP9 was prominently active in PC3 cells. Thus we set out to test the possible role of MMP9 in mediating the effects of PDEF on cell invasion. For these studies we evaluated the effects of PDEF expression on MMP9 mRNA expression, promoter activity and enzymatic activity. As can be seen in Figure 4B &4C, PDEF expression completely abolished MMP9 mRNA expression and enzymatic activity, and significantly reduced MMP9 promoter activity in PC3 cells compared to vector control. These data demonstrate inhibition of MMP9 expression by PDEF, and for the first time demonstrate regulation of MMP9 by any ETS transcription factors. To further confirm the role of MMP9 in modulating invasive behavior of prostate cancer cells, we performed antibody-neutralizing experiments. For these studies, we added MMP9 antibodies to the cells during the invasion assay, and data showed that anti MMP9 antibody inhibited cell invasion in PC3 cells by ~70% as compared to control IgG (Figure. 4D), further supporting the role of MMP9 in mediating the invasive phenotype in prostate cancer cells. Taken together these results demonstrate that PDEF negatively regulates MMP9 expression and provide a possible mechanism of PDEF actions in suppression of the invasive phenotype in prostate cancer.

### PDEF expression in metastatic Prostate cancer cells results in phenotypic reversal and decreased migration in three dimensional cultures

To examine the effects of PDEF expression in a context that more closely resembled *in vivo *settings, we assessed the consequence of PDEF expression in PC3 cells on acinar or spheroid formation in 3 D culture. Results presented in Figure 5 demonstrate that PDEF expressing PC3 cells formed spheroid-like structures in basement membrane cultures, while most of the vector control cells form irregular structures and projections emanating from these structures that readily migrated and invaded the basement membrane by 10-12 days of culture. Several recent studies demonstrated inverse relationship between spheroid formation with cell migration and invasion. Our results show that re-introduction of PDEF in PC3 cells resulted in re-establishment of cellular polarity leading to inhibition of cell migration and reversal to less invasive phenotypes.

**Figure 5:** **Effect of PDEF expression on cells grown in three dimensional cultures**. ***A***, representative images of three dimensional matrigel culture of PC3 cells with and without PDEF showing phenotypic reversal. Representative phase image obtained at various days in culture using 20X objective. ***B*, Fluorescence **microscopic images of PDEF PC3 cells and vector control cells after phalloidin and DAPI staining in 3 D cultures. **C**) Schematic depiction of the effects of PDEF expression in Prostate cancer cells.

### Phosphorylation of PDEF and PDEF T50A

Since the T50A mutant had little or no effect on many of the phenotypic features associated with aggressive behavior, we asked whether the T50 phosphorylation site was a major contributor to PDEF phosphorylation. PC3 cells were transiently transfected with PDEF, the T50A mutant, or empty vector, and labeled with ^32^P-phosphoric acid. FLAG-PDEF immunoprecipitates were sequentially analyzed by autoradiography and Western blotting. The results (Figure S3, Additional file 1) indicate that PDEF T50A is phosphorylated, suggesting that amino acids other than T50 in the protein are kinase targets. Of interest, we found in this experiment that elimination of reducing agents during electrophoresis resulted in an approximate doubling of PDEF's apparent molecular weight (under reducing conditions about 45 kd), suggesting that native PDEF exists as a disulfide complex with another molecule(s). Overall, these findings suggest that amino acids other than the MAPK phospho-acceptor site at T50 in the protein could be possible targets for kinase, and they might have essential regulatory mechanism for invasion and migration. Thus, the T50A mutation does not alter the functions of PDEF and PC3 cells can phosphorylate PDEF at other locations.

### MMP9 expression is increased in progression from normal to high grade prostate carcinomas and is inversely associated with PDEF expression

To further test whether MMP9 expression correlated with aggressive behavior of prostate cancer cells and to test whether a correlation existed between MMP9 and PDEF expression in human prostate cancer specimens, we evaluated MMP9 expression in the same tissue microarray slides containing 40 cores of prostate cancer and 9 cores of normal prostate that were used for PDEF expression analysis. Results presented in Figure 6A &6B show that MMP9 expression is up-regulated during the transition to high grade prostate cancer. Results presented in Figure. 6B, demonstrate that MMP9 protein staining was observed predominantly (>60-80%) in high grade prostate cancer cells (Gleason 8, 9 & 10), whereas normal prostate cells had very little or undetectable levels of MMP9 protein. Increased MMP9 protein expression was observed in 38 cores of prostate tumor tissue whereas 2 cores of prostate cancer had no positive staining for MMP9. For low grade prostate cancer (Gleason 7 or below) 21 ± 3% tissue scored positive for MMP9 (staining >40-80%) whereas for Gleason 8 to 10 it increased to 60 ± 9.3%. Combining all, these results indicate that there is significant co-relation between the low MMP9 expression in normal tissue with high MMP9 in intermediate to high Gleason prostate carcinoma.

**Figure 6:** **MMP9 protein expression in Human prostate tissues**. ***A***, Immunohistochemistry for Representative photo-micrographs of Immuno-histochemical analysis of MMP9 expression using prostate tissue micro-array slides (containing both normal and tumor samples of different grades) performed as described in Materials and Methods. ***B***, Quantification of percentage staining for MMP9.

### Inverse relationship between PDEF and MMP9 expression in human prostate tissue

Our analysis of the PDEF and MMP 9 protein expression data presented in Figure 1 and 6 revealed that in human prostate tissue PDEF levels were lower in tumor samples as compared to normal tissue, however this difference reached a statistical significance only in prostate cancer samples form Gleason 8 and above (Normal vs. Gleason 6 & 7 Grade: p = 0.3593; Normal vs. Gleason 8 Grade: p = 0.0176; Normal vs. Gleason 9 & 10 Grade: p < 0.001). By contrast, we observed that MMP9 levels were higher in tumor samples as compared to normal tissue. Again the difference in MMP9 expression reached statistical significance only in prostate cancer samples form Gleason 8 and above (Normal vs. Gleason 6 & 7 Grade: p = 0.1517; Normal vs. Gleason 8 Grade: p = 0.0076; Normal vs. Gleason 9 & 10 Grade: p < 0.001). These data are presented for each individual sample in Figure 7A.

**Figure 7:** **Relationship between PDEF and MMP9 expression in human prostate tissue: ***A***, Expression of PDEF and MMP9 in individual samples B) Regression plot of the data presented in A**. Data were collected from the immunohistochemistry performed for PDEF and MMP9 as described for Figure 1 and 6. (Normal = red; Gleason 6 & 7 = blue; Gleason 8 = green; and Gleason 9 and 10 = black). By regression analysis, there is a significant 0.846 (UNITS) drop in MMP9 for every 1.0 (UNIT) increase in PDEF.

Our regression analyses of these data reveal an inverse correlation between PDEF and MMP9 levels (Figure 7B and Table S1, Additional file 1). Thus, a decreased expression of PDEF in prostate cancer is associated with the malignant phenotype, more aggressive tumor behavior, and increased MMP9 expression.

## Discussion

This is the first study to demonstrate loss of PDEF protein expression in high grade prostate cancer as compared to normal prostate as well as low grade prostate cancer tissue; and phenotypic reversal of highly migratory, invasive and aggressive prostate cancer cells to adherent polarized and non invasive cells in three dimensional cultures upon re-introduction of PDEF. We also show for the first time regulation of MMP9 by PDEF, and a direct correlation between loss of PDEF and increased expression of MMP9 high grade prostate cancer.

The ETS family is one of the largest families of transcription factors with 27 genes in human chromosome. The ETS family is present throughout the body and is involved in a wide variety of functions including the regulation of cellular differentiation, cell cycle control, cell migration, cell proliferation, apoptosis (programmed cell death) and angiogenesis. Multiple Ets factors have been found to be associated with cancer, such as through gene fusion including prostate cancer (2, 20-25). PDEF is selectively localized to the tissues with high epithelial content including prostate, and like other Ets family members has been shown to have diverse biological functions including tumor suppressor as well as tumor promoter functions.

Our results demonstrate loss of PDEF in high grade prostate cancer as compared to low grade prostate cancer as well as normal prostate tissue. Our results are unique in a way that they demonstrate for the first time loss of PDEF is associated with aggressive phenotype in prostate cancer, and suggest that PDEF might serve as a potential marker for distinguishing aggressive prostate cancer from an indolent disease. These findings are in apparent contrast to the previously published studies that concluded over expression of PDEF in prostate cancer as compared to normal prostate tissue [11]. It is important to point out here that previous studies lumped together all cancer samples and compared them with normal tissue, however, they did not attempt subset analysis of PDEF expression between low grade and high grade disease, which could have resulted in different conclusions. Our conclusion that PDEF expression is a favorable indicator in prostate cancer is, however, in agreement with studies that demonstrated a positive prognostic value of PDEF in ovarian cancer[8].

Our results also show that re-introduction of PDEF in aggressive prostate cancer cells resulted in decreased cell migration, decreased directional migration as well as decrease in clonogenic activity and converse was true when we knocked down PDEF in prostate cancer cells expressing PDEF (Figure S2, Additional file 1). These data suggest PDEF might serve as a suppressor of tumor migration and clonogenic activity. These results are in agreement with the previous studies with various breast and prostate cancer cells [5,7]. Our results are, however in sharp disagreement with studies that suggested that PDEF might promote migratory phenotype in breast cancer cells [3].

In order to become motile, cancer cells establish a defined polarity in the direction of movement through interaction between lamellipodia (a cytoskeletal actin projection on mobile edge of the cells) and focal adhesions that facilitate adhesion and migration of the cells. We also observed distinct changes in cytoskeleton and cell morphology associated with PDEF expression. We also show for the first time in any system that that PDEF expression increased cell adhesion, and resulted in a significant reduction in FAK phosphorylation. In previous studies we have shown an essential role for FAK in aggressive phenotype in prostate cancer cells [19]. Thus modulation of cytoskeleton organization and FAK activity by PDEF expression may provide potential pathways by which PDEF modulates cell behavior. These results extend previous observations in several cell types that show SiRNA mediated knockdown of PDEF was associated with increased cell migration [3-5]. While the results discussed so far point to the possible role of PDEF expression in modulating phenotypic behavior of cancer cells, our studies, are the first to use three dimensional cultures to actually demonstrate directly the effects of PDEF on cellular polarity and spheroid formation. Results clearly demonstrate that re-introduction of PDEF in aggressive prostate cancer cells resulted in phenotypic reversal from a disorganized, migratory and invasive cell growth to an organized, non-migratory and non-invasive phenotype.

Chintala et al. reported that the formation of spheroids is also linked to reduced invasion and expression and activity of MMP9 [26]. Matrix metalloproteinases (MMP) are a family of enzymes whose function primarily relates to the degradation of extracellular matrix proteins, and which are necessary for cell invasion. Our results presented here show that upon PDEF expression, prostate cancer cells lose their ability to invade Matrigel in Boyden chamber assays. These results are similar to the results observed by Turner et al. in invasive breast cancer cells [4]. However, to the best of our knowledge, our results show for the first time that PDEF downregulates MMP9 expression, and its promoter activity in any cell type. We observed that expression of PDEF in PC3 cells resulted in loss of MMP9 mRNA expression, decrease in MMP9 promoter activity and a significant reduction in the gelatinolytic activity. Thus our results again highlight a unique property of PDEF that is distinct from other ETS factors. We carried out additional studies to directly evaluate the functional consequence of MMP9 activity in PC3 cells. Results of these studies demonstrate that antibody mediated neutralization of MMP 9 reduced the invasion of PC3 cells through basement membrane matrix similar to that observed upon PDEF expression. Overall these findings provide for a mechanism by which PDEF expression could modulate cell polarity and other aggressive behavior.

Since we observed negative regulation of MMP9 by PDEF and published results suggested that the activity of MMP9 is associated with the progression and metastasis of prostate cancer [27], we also evaluated MMP9 expression in the tissue microarray slides containing 40 cores of prostate cancer and 9 cores of normal prostate that were used for PDEF expression analysis. Our results demonstrated an increase in MMP9 expression in high grade prostate cancer, which is in agreement with the previous studies [27]. We also observed an inverse correlation between PDEF expression and MMP9 expression in these samples. These results are in agreement with our findings in tissue culture studies that demonstrated negative regulation of MMP9 expression by PDEF. These results also highlight the potential use of loss of PDEF expression and increased MMP9 expression in early detection of aggressive prostate cancer.

## Conclusions

In summary results presented herein demonstrate for the first time that PDEF, a member of Ets family, is lost in high grade prostate cancer and decreased PDEF expression is associated with increased MMP9 expression. We also provide direct evidence for the first time demonstrating that PDEF expression results in phenotypic reversal of aggressive prostate cancer cells in three dimensional cultures. Our studies also provide first demonstration in any system of negative regulation of MMP9 expression by PDEF. Taken together, our studies suggest that PDEF, by virtue of suppressing MMP9 expression and by modulating the ability of cancer cells to form a temporal structure required for migration and invasion, may function as suppressor of tumor metastasis in prostate cancer and perhaps other cancers. Our observation of an inverse relationship between PDEF and MMP9 expression suggests that expression of PDEF along with decreased MMP9 could help in early detection of aggressive prostate cancer and may facilitate new approaches to prostate cancer treatment.

## Competing interests

A patent application relating in part to the content of the manuscript is being prepared.

No other interests

## Authors' contributions

HKK designed research; TJ cloned PDEF, made stable cell lines and performed most of the cell migration, adhesion and invasion assays; S.K. performed all of the experiments with PDEF and MMP 9 expression in clinical samples and MMP 9 gene expression in cell lines. BK performed 3 D culture assays, cytoskeleton imaging, zymograms and the MMP 9 antibody neutralization assays; LK performed phospho-FAK assays and helped with cell culture work; SV performed many colony formation assays and assisted in the retrovirus and cloning work; TJ, BK, SK, PM, RBM and HKK analyzed data; and BK, TJ, LK, SK and HKK wrote the paper. All authors read and approved the final manuscript.

## Supplementary Material

Additional File 1 **Supplementary data**. Supporting Information. Materials and Methods with respect to following: -Immunofluorescence of cultured cells. -Anchorage independent Growth, and invasion assays. -Western blot analysis. -Metabolic Labeling. Figure S1 PDEF expression in cultured cells with or without PDEF. Figure S2 PDEF knockout increased colony formation and invasion of LNCaP and LNCaP C4-2B cells. Figure S3 Phosphorylation of PDEF and PDEF T50A. Table S1 Relative PDEF and MMP9 gene expression in human prostate tissue. Click here for file
